This article has been retracted.

# Preoperative Nutritional Status and Risk Factors Associated with Delayed Discharge in Geriatric Patients Undergoing Gastrectomy: A Single-Center Retrospective Study

**DOI:** 10.1155/2022/8263986

**Published:** 2022-06-03

**Authors:** Xining Zhao, Jie Liu, Ying Wang, Yuying Yang, Yan Pan, Shengjin Ge

**Affiliations:** Department of Anesthesiology, Zhongshan Hospital Fudan University, Shanghai 200032, China

## Abstract

**Objective:**

Preoperative malnutrition is an independent risk factor for postoperative complications and survival for gastric cancer patients. The study is aimed at investigating the prevalence of malnutrition, perioperative nutritional support, and the risk factors associated with delayed discharge of geriatric patients undergoing gastrectomy.

**Methods:**

A retrospective study of gastric cancer patients (age ≥ 65) who underwent gastrectomy at Zhongshan Hospital from January 2018 to May 2020 was conducted. Clinical data, including demographic information, medical history, surgery-related factors, and perioperative nutritional management, were collected and analyzed. Postoperative complications were assessed according to the Clavien-Dindo grading system, and the prognostic nutritional index (PNI) was calculated. The risk factors affecting the prolongation of postoperative hospital stay were analyzed.

**Results:**

A total of 783 patients were reviewed. The overall frequency of malnutrition was 31.3% (249/783). The albumin, prealbumin, and hemoglobin levels were lower in the malnutrition group than in the well-nourished group. The proportion of patients who received preoperative total parenteral nutritional support in the malnutrition group was significantly higher than in the well-nourished group (12.4% vs. 3.7%, *P* < 0.001). All patients received postoperative parenteral nutrition (PN); the proportion of patients who received total nutrient admixture (TNA) in the malnutrition group was lower than in the well-nourished group (22.1% vs. 33.5%, *P* = 0.001). No significant difference was found in the duration of postoperative nutrition between groups (*P* > 0.05). The malnutrition group was associated with a higher rate of postoperative complications (*P* < 0.001). Univariate and multivariate regressions revealed that age > 70 years (OR = 1.216, 95% CI 1.048-1.411, *P* = 0.010), operation time > 180 min (OR = 1.431, 95% CI 1.237-1.656, *P* < 0.001), PNI < 44.5 (OR = 1.792, 95% CI 1.058-3.032, *P* = 0.030), and postoperative complications (OR = 2.191, 95% CI 1.604-2.991, *P* < 0.001) were significant risk factors associated with delayed discharge.

**Conclusion:**

Malnutrition is relatively common in elderly patients undergoing gastrectomy. Advanced age, duration of surgery, lower levels of PNI, and postoperative complications were risk factors associated with delay discharge. Elderly gastric cancer patients with risk factors urgently require specific attention for reducing hospital stay.

## 1. Introduction

Gastric cancer (GC) remains the 5^th^ most common cancer worldwide [1] and had the second-highest mortality rate in China [2]. The population of elder patients with GC has been increasing because of the high prevalence of *H. pylori* infection and increasing life expectancy. Elderly GC patients face several challenges during treatment, such as comorbidities, organ dysfunction, immunosuppression, and delayed recovery [3, 4]. Advanced age is associated with a higher rate of postoperative complications shortly after surgical treatment [5] and lower 5-year overall survival as long-term outcome [6].

In China, the prevalence of malnutrition in hospitalized patients is around 12.6% to 46.19% [7–10]. Malnutrition is one of the great risk factors of adverse clinical outcomes in elderly patients with GC [11]. The nutritional status at the time of diagnosis was independently associated with postoperative complications, overall survival, and disease-free survival [12, 13]. The condition can be caused by mechanical obstruction of the digestive tract or anorexia-cachexia syndrome, leading to insufficient protein or energy intake and absorption disorder. Nutrition screening, assessment, and intervention are important steps in nutritional management.

Previous studies mostly focused on hospitalized internal medical patients [14]. Only a few studies focused on surgical patients regardless of age [9]. Therefore, in this retrospective study, we investigated the nutritional status and perioperative nutritional support of geriatric surgical patients with GC and provide a basis for implementing an effective nutritional intervention.

## 2. Methods

### 2.1. Study Design and Participants

The research project was a retrospective, observational study approved by the Ethics Committee of Zhongshan Hospital (B2021-392) and was conducted in accordance with the Declaration of Helsinki. The records of elderly patients with GC who underwent open gastrectomy and were 65 or older between May 2018 and May 2021 at Zhongshan Hospital affiliated to Fudan University were retrospectively identified. Patients with other malignancies, previous gastrointestinal surgery, emergency surgery, or incomplete medical record were excluded.

Clinical data, including demographic information, medical history, laboratory tests, postoperative complications, lengths of hospital stay (LOS), and cost were collected and analyzed. Postoperative complications (PPC) were graded according to the Clavien-Dindo (CD) classification [15], and grade II or higher were regarded as complications [16].

### 2.2. Definition and Assessment of Malnourished Patients

Malnutrition was defined, according to the European Society for Clinical Nutrition and Metabolism (ESPEN) diagnostic criteria [17], as a weight loss of more than 10% (indefinite of time) or more than 5% over the last 3 months and a body mass index (BMI) < 20 kg/m^2^ or <22 kg/m^2^ in patients under or above the age of 70, respectively. Nutritional assessment was performed based on a prognostic nutritional index (PNI), which is an easily available index widely employed for evaluating the nutritional status of patients with gastric cancer [18]. The PNI was calculated based on the equation: [(10 × serum albumin (g/dL)) + (0.005 × total lymphocyte count (/mm^3^))]. The composition and duration of nutritional management were recorded and analyzed.

### 2.3. Statistical Analysis

All statistical analyses were performed using SPSS ver. 22.0 (IBM SPSS, Chicago, USA). Normal distribution measurement data were expressed as mean ± SD, and *t*-test was used to compare the differences between the groups. The measurement data of skewed distribution were expressed as median (interquartile range), and the categorical variables were expressed as counts and percentages and compared using the *χ*^2^ test. Univariate and multivariate analyses were carried out using logistic regression. The *P* value was considered to be statistically significant at 0.05 level.

## 3. Results

### 3.1. General Characteristics

A total of 783 adults were included in this study (Figure 1). The characteristics of the patients were shown in Table 1. The median age at diagnosis was 70 years (range: 65-86 years). The proportion of male individuals was 584 (74.6%). Among the 783 individuals, 76 (9.7%) suffered from 3 or more chronic diseases. There were 132 (16.9%) patients received preoperative consultation because of comorbidities.

### 3.2. Malnutrition

The frequency of malnutrition is shown in Table 1. The overall frequency of malnutrition was 31.8%. The age in the malnourished group (M group) was significantly higher than that in the well-nourished group (W group) (72 vs. 69, *P* < 0.001). Significant differences were found in albumin, prealbumin, hemoglobin, and PNI between the M group and W group (*P* < 0.05). The number of patients with 3 or more preoperative comorbidities, gender ratio, surgery type, surgery time, anesthetic method, preoperative consultation, and preoperative neoadjuvant therapy was of no significance between the two groups (*P* > 0.05).

### 3.3. Preoperative Nutritional Support

As shown in Table 2, of the 783 elderly individuals, 424 (54.1%) received nutritional support. Of the 249 elderly patients with malnutrition, 77 (30.8%) received a single nutritional transfusion and 31 (12.4%) received total parenteral nutrition (TPN). Of the 534 individuals without malnutrition, 296 (55.4%) received a single transfusion and 20 (3.7%) received TPN. The composition of nutritional support was mainly carbohydrates based on diet. The rate of TPN was higher in the M group than in the W group (*P* < 0.001).

### 3.4. Postoperative Nutritional Support

All patients received parenteral nutrition after surgery. Of the 249 malnutrition patients, 194 (77.9%) patients were given a single transfusion of carbohydrates with or without composite amino acid, and 55 (22.1%) received total nutrient admixture (TNA). In patients with normal nutrition, 355 (66.5%) received single transfusion and 179 (33.5%) received TNA. The proportion of patients in the M group who received TNA was significantly lower than that in the W group (*P* = 0.001). No significant differences were found in rates or duration of postoperative nutrition between the two groups (*P* > 0.05) (Table 2).

### 3.5. Postoperative Complications

Comparing the two groups, the incidence of PPC in group M was significantly higher than that in group W (grade I-II: 10.8% vs. 6.9%; grade III-V: 11.6% vs. 3.9%; *P* < 0.001). There was no significant difference in hospital mortality, unplanned readmission rate within 30 days, LOS, and cost between the two groups (*P* > 0.05) (Table 2).

### 3.6. Risk Factors Associated with Prolonged LOS

The median LOS was 8 d (Table 2); therefore, a LOS of 9 d or more was defined as prolonged LOS. Factors such as patient age, gender, nutritional status, operation time, anesthesia method, chronic comorbidities, postoperative nutritional support, and PPC were included in the univariate analysis. Age ≥ 70 years, operation time ≥ 180 min, PNI < 44.5, and CD ≥ 3 were related factors of prolonged LOS (*P* < 0.05). The factors with *P* > 0.1 in the univariate analysis were used as independent variables, and the occurrence of prolonged LOS was used as the dependent variable. The multivariate logistic regression showed that age ≥ 70 years (OR = 1.216, 95% CI 1.048-1.411, *P* = 0.010), operation time ≥ 180 min (OR = 1.431, 95% CI 1.237-1.656, *P* < 0.001), PNI < 44.5 (OR = 1.792, 95% CI 1.058-3.032, *P* = 0.030), and CD grade I-II (OR = 2.191, 95% CI 1.604-2.991, *P* < 0.001) (Table 3).

## 4. Discussion

In the present study, the prevalence of preoperative malnutrition in elderly patients undergoing gastrectomy was 31.3%, which was relatively high compared with that in previous studies [9]. Many factors are contributed to observed differences in malnutrition prevalence include instruments, age distribution, hospital location, and characteristics of the patients. Patients with preoperative malnutrition were associated with low levels of albumin, prealbumin, and hemoglobin than well-nourished patients. Furthermore, malnourished elderly patients were found to be associated with higher postoperative complications and prolonged length of hospital stay than well-nourished elderly. There was no significant difference in composition and timing of postoperative nutritional management between malnourished and well-nourished patients.

Malnutrition is one of the risk factors for PPC [19]. In old patients with GC, malnutrition is often caused by frailty, absorption disorder, and a decrease in food intake [20]. These patients often develop anemia, hypoproteinemia, and electrolyte abnormalities before surgery. Therefore, screening and assessing for malnutrition is an important step for all patients scheduled for major gastrointestinal surgery. The preoperative PNI is an independent prognostic factor for disease-free along with age and TNM stage in GC patients after surgery [21]. A recent study found that preoperative PNI is a sensitive and specific prognostic predictor among elderly patients undergoing gastric cancer surgery [22]. The result in our study showed that low PNI is an independent risk factor associated with prolonged LOS, suggesting that PNI is a predictor for both short-term and long-term outcomes for elderly patients. Meantime, the measurement of PNI (albumin and lymphocyte count) is simple and convenient to achieve.

The guidelines of both the American Society for Parenteral and Enteral Nutrition (ASPEN) and the ESPEN recommend oral or enteral feeding whenever possible [23, 24]. Enteral nutrition is preferred over parenteral nutrition because of a lower incidence of surgical site infection [25]. But in patients with a pyloric obstruction or inadequate energy supply by enteral nutrition, peripheral parenteral nutrition or TPN is often performed [23]. In our study, the rate of preoperative TPN in patients with malnutrition was significantly higher than in well-nourished patients. However, the total rate of preoperative parenteral nutrition support was still low (43.5%) in patients with malnutrition. Optimal preoperative management for elder patients with malnutrition is essential to improve surgical outcomes.

Although early initiation of oral or enteral feeding has been recommended to improve clinical outcomes and to reduce surgical complications in GC patients following gastrectomy [23, 26], the postoperative nutritional support for patients is quite variable between different surgical teams. And in the statement of the Japanese Gastric Cancer Treatment Guideline, the drink should be offered after postoperative day 1 and a solid diet should begin from postoperative day 2 to 4 regardless of surgery type [27]. In this study, the median period of parenteral nutrition is 5 days. Meanwhile, 54.8% of old patients received only carbohydrates with or without composite amino acids postoperatively. No significant difference was found in duration between malnourished and well-nourished patients. It might take some time before patients with malnutrition are properly taken in charge. This study also supported the findings of previous studies that patients with malnutrition have a higher rate of overall postoperative complications [19, 28]. This indicated that old patients with malnutrition should be paid more attention during the postoperative period, and nutritional support should be individualized for these vulnerable patients.

At multivariate analysis, we found that longer duration of surgery was significantly related with delayed discharge, which was in accordance with previous study [29]. This suggested that the length of surgery could be regarded as a convenient marker of surgical stress burden, and patients going through a long period of surgery need special care postoperatively.

The novelty of this study was the assessment of nutritional status and risk factors associated with delayed discharge among geriatric GC patients with a large sample size in China. As a single-center retrospective study, this study had several limitations. We did not follow up for long-term outcomes, and we could not investigate the relationship between perioperative nutritional support and clinical outcomes among malnourished patients. Therefore, large multicenter prospective RCTs should be conducted to further investigation.

## 5. Conclusion

In conclusion, malnutrition is relatively common in elderly patients undergoing gastrectomy. Age, length of surgery, PNI, and postoperative complications were risk factors associated with delay discharge. Elderly gastric cancer patients with risk factors urgently require specific attention for reducing hospital stay.

## Figures and Tables

**Figure 1:** Flowchart of patients' selection.

**Table 1:** Clinical and nutritional characteristics of malnourished and well-nourished elderly patients.

Item	Group	All (*n* = 783)	Malnourished (*n* = 249, 31.8%)	Well-nourished (*n* = 534, 68.2%)	*t*/*χ*^2^/*F*	*P*
Age, years	Median (IQR)	70 (67, 74)	72 (69, 76)	69 (67, 73)	36.700	<0.001
Gender, *n* (%)	Male	584 (74.6)	184 (74.9)	400 (73.9)	0.092	0.762
	Female	199 (25.4)	65 (25.1)	134 (26.1)		
BMI (kg/m^2^)		22.9 ± 3.4	19.4 ± 1.8	24.5 ± 2.6	-31.949	<0.001
Number of chronic diseases, *n* (%)	0 ~ 2	707 (90.3)	221 (88.8)	486 (91.0)	0.986	0.321
	≥3	76 (9.7)	28 (11.2)	48 (9.0)		
PNI		48.1 ± 5.6	48.8 ± 5.3	46.7 ± 5.7	-5.108	<0.001
Albumin (g/L)		40.2 ± 4.3	39.1 ± 4.6	40.7 ± 4.0	-4.680	<0.001
Prealbumin (mg/L)		207.8 ± 49.6	193.2 ± 50.6	214.6 ± 47.7	-5.709	<0.001
Hemoglobin (g/L)		121.0 ± 23.6	117.0 ± 24.1	122.8 ± 23.1	-3.205	0.001
TLC (×10^9^/L)		1.59 ± 0.54	1.57 ± 0.55	1.60 ± 0.54	0.719	0.472
Type of surgery, *n* (%)	Total gastrectomy	359 (45.8)	112 (45.0)	247 (46.3)	0.653	0.721
	Distal gastrectomy	397 (50.7)	130 (52.2)	267 (50.0)		
	Proximal gastrectomy	27 (3.4)	7 (2.8)	20 (3.7)		
Operation time (min)	Median (IQR)	160 (123, 189.5)	160 (126, 189)	160 (129, 191)	3.025	0.082
Type of anesthesia, *n* (%)	GA	87 (11.1)	35 (14.1)	52 (9.7)	3.206	0.073
	TEA	696 (88.9)	214 (85.9)	482 (90.3)		
Preoperative consultation, *n* (%)	Yes	132 (16.9)	47 (18.9)	85 (15.9)	1.060	0.303
	No	651 (83.1)	202 (81.1)	449 (84.1)		
Preoperative neoadjuvant chemotherapy, *n* (%)	Yes	25 (3.2)	9 (3.6)	16 (3.0)	0.210	0.647
	No	758 (96.8)	240 (96.4)	518 (97.0)		
Tumor stage, *n* (%)	I	126 (16.1)	32 (13.0)	87 (16.2)	7.452	0.059
	II	150 (19.2)	53 (21.3)	133 (24.9)		
	III	402 (51.3)	128 (51.3)	267 (50.0)		
	IV	105 (13.4)	36 (14.4)	47 (8.9)		

Abbreviations: BMI: body mass index; PNI: prognostic nutritional index; TLC: total lymphocyte count; GA: general anesthesia; TEA: general anesthesia combined with thoracic epidural block.

**Table 2:** Preoperative and postoperative nutritional supports among elderly gastric cancer patients with or without malnutrition.

		All (*n* = 783)	Malnourished (*n* = 249, 31.8%)	Well-nourished (*n* = 534, 68.2%)	*Z*/*χ*^2^/*F*	*P*
Preoperative nutrition, *n* (%)	Diet	359 (45.9)	141 (56.6)	218 (40.8)	14.75	<0.001
	Diet+single transfusion	373 (47.6)	77 (30.8)	296 (55.4)		
	TPN	51 (6.5)	31 (12.4)	20 (3.7)		
Postoperative nutrition, *n* (%)	Single transfusion	549 (70.1)	194 (77.9)	355 (66.5)	10.592	0.001
	TNA	234 (29.9)	55 (22.1)	179 (33.5)		
PN period	Median (IQR), day	5 (4, 6)	5 (4, 6)	5 (4, 6)	0.004	0.951
EN period	Median (IQR), day	2 (1, 2)	2 (1, 3)	2 (1, 2)	1.201	0.273
Clavien-Dindo grade	No, *n* (%)	669 (85.4)	193 (77.5)	476 (89.1)	21.696	<0.001
	I-II, *n* (%)	64 (8.2)	27 (10.8)	37 (6.9)		
	III or higher, *n* (%)	50 (6.4)	29 (11.6)	21 (3.9)		
In-hospital mortality	n	2	2	1		0.535
Readmission within 30 d	n	15	11	4		0.79
Length of hospital stay	Median (IQR), day	8 (7, 10)	8 (7, 9)	8 (7, 10)	-1.504	0.133
Cost of hospitalization	Median (IQR), K¥	54.8 (47.7, 64.7)	55.3 (47.4, 66.6)	54.7 (47.8, 63.2)	-1.051	0.293

Abbreviations: EN: enteral nutrition; PN: parenteral nutrition; TPN: total parenteral nutrition; TNA: total nutrient admixture; IQR: interquartile range. The “¥” refers to RMB, and “K¥” refers to "per 1000 RMB".

**Table 3:** Univariate and multivariate analyses of clinical factors associated with prolonged length of stay.

Clinical factors	Group	*N* = 783	LOS	Univariate analysis		Multivariate analysis		
			(days)	*χ* ^2^	*P*	OR	95% CI	*P*
Sex	Male	584	8 (7, 10)					
	Female	199	7 (7, 9)	3.142	0.076	0.962	(0.817, 1.132)	0.637
Age (years)	65~70	349	7 (7, 9)					
	≥70	434	8 (7, 10)	9.730	0.002	1.216	(1.048, 1.411)	0.010
Nutritional status	Well-nourished	534	8 (7, 9)					
	Malnourished	249	8 (7, 10)	2.245	0.134	0.990	(0.842, 1.163)	0.899
Surgery time (min)	<180	438	7 (7, 8)					
	≥180	345	8 (7, 11)	44.218	<0.001	1.431	(1.237, 1.656)	<0.001
Anesthesia	GA	87	8 (7, 11)					
	TEA	696	8 (7, 9)	2.714	0.099	0.921	(0.734, 1.154)	0.474
Comorbidity	<3	707	8 (7, 9)					
	≥3	76	8 (7, 11)	3.915	0.048	1.067	(0.839, 1.357)	0.595
Hemoglobin (g/L)	≥90	675	8 (7, 9)					
	<90	108	8 (7, 11)	1.893	0.169			
Albumin (g/L)	>30	772	8 (7, 9)					
	≤30	11	10 (7, 11)	1.789	0.181			
Prealbumin (mg/L)	≥180	523	8 (7, 9)					
	<180	260	8 (7, 10)	7.389	0.007	0.797	(0.514, 1.237)	0.312
Postoperative PN	Single transfusion	549	8 (7, 10)					
	TNA	234	8 (7, 9)	0.317	0.573			
PNI	≥44.5	718	8 (7, 11)					
	<44.5	65	9 (8, 13)	7.856	0.005	1.792	(1.058, 3.032)	0.030
Clavien-Dindo grade	0	669	8 (7, 9)					
	1 ~ 2	64	10 (7, 12)			2.191	(1.604, 2.991)	<0.001
	≥3	50	10 (7, 17)	40.624	<0.001	1.163	(1.163, 1.701)	0.435

Abbreviations: LOS: length of stay; GA: general anesthesia; TEA: general anesthesia combined with thoracic epidural block; PN: parenteral nutrition; TNA: total nutrient admixture; PNI: prognostic nutritional index.

## Data Availability

The data used to support the findings of this study are available from the corresponding author upon request.
